# Optimization of Thumb Prosthesis Design by Using Five Performance Criteria

**DOI:** 10.1155/2022/9647956

**Published:** 2022-09-05

**Authors:** Nestor Tsamo, Denis Tcheukam Toko, Pierre Kisito Talla

**Affiliations:** ^1^Laboratory of Mechanics and Modelling of Physical Systems (L2MPS), Department of Physics, Faculty of Science, University of Dschang, P. O. Box: 67, Dschang, Cameroon; ^2^Mechanical Engineering Department, College of Technology, University of Buea, P.O. Box 63 Buea, Cameroon

## Abstract

The thumb prosthesis mechanism is optimally designed by using five performance criteria including the following: least square structural error, mechanical manufacturing imprecision error, driving optimal torque, mechanical strength reliability, and production cost of the thumb mechanism. This paper was devoted to the optimization of the thumb prosthesis's mechanism by taking into consideration the manufacturing cost model based on machining cost theory which took into detail the shape of the workpieces and the strength reliability of all the parts composing the entire mechanism. Every optimization problem displays a particular set of an independent vector of optimal parameters, showing the impact of each objective function on the configuration of the prosthetic device. The multiobjective optimization showed that the mechanical reliability and the production cost included in any combination of the simultaneous optimization enabled the achievement of the same optimum variables design, though with some exceptions. With the inclusion of the labor charges, the depreciation rate of the equipment, and production assets in the mathematical's manufacturing cost model, the optimal manufacturing cost generated from the numerical simulation was 501.0021 USD. Therefore, the global manufacturing cost and the mechanical strength reliability of the whole prosthesis mechanism have a real impact on the customization of the structure, due to the stochastic nature of the trajectory of the cutting tools during the manufacturing processes.

## 1. Introduction

The invention of new prosthetic devices over the past decades has observed advances as a consequence of recent technological development, advancing in the aspect of greater dexterous hand devices. The use of a mechanical prosthesis to replace a missing limb is one of the most fascinating challenges faced by prosthetists in the prosthetic rehabilitation protocol [1–4]. The level of autonomy and the capabilities of performing social activities, trade, and daily tasks negatively influenced amputees. However, the state-of-the-art prosthesis failed to coalesce smooth functioning, reliability, suitable personalized aesthetic, adequate maintenance, affordability, and sometimes adequate grasping [5, 6]. Most prostheses fail to closely match the user-specific requirement and have poor design, resulting in the abandonment of the artificial device by the amputees [7]. One of the most popular works on prosthesis optimization in the literature has been done by Vinet et al. [8]. They obtained all the bending angles of the hand morphology using 3D graphical software CATIA on four planar bar mechanisms.

The thumb plays a paramount role in the various grasping modes. Liken to unfavorable conditions such as sickness, accident, or congenital malformation, the rehabilitation process of the thumb is greatly affected especially by its contribution to six grasping modes retained by many prosthetists [9, 10]. The design of a thumb prosthetic device is critical since forty percent of the entire functionality of the human depends on the hand. In housekeeping and laundry, the grasping mode is dominated at sixty percent by the contribution of the thumb. Many prosthetists faced the challenge to choose a simple, accurate, and less mobility or degree of freedom, which allows equal force distribution. The least square structural error on the second phalanx of the thumb and the trajectory of the model is determined by the end reflector which is the fingertip [11, 12]. To obtain the safe, smooth, accurate, and affordable functionality of the thumb, one of the most interesting solutions is the use of the planar articulated crossed four-bar mechanism to design the prosthetic mechanism as shown in Figure 1. The synthesis followed by the design methodology of mechanisms has been the subject of several investigations [1–4, 8, 13].

The main objective of this paper is to introduce into upper limb optimization processes the mechanical reliability of each element of the basic mechanism, used to design the artificial device. Their applications are numerous and their synthesis is generally done by reference to *n* input positions and *n* output positions of the considered parameters [14]. The four-link articulated planar mechanism proposed for synthesis finds application in a hand prosthesis that can perform various types of grasping daily objects. Its optimal synthesis will be made by reference to *n* positions of the coupling and output members. For this purpose, two performance criteria are used: the least square structural error on the angle of flexion of the second phalanx of a thumb and the maximum motor torque necessary to balance a given force at the tip of this finger. This paper will also integrate the global manufacturing cost model taking into account the stochastic nature of the trajectory of the cutting tools during the machining process on the numerical control machine center. This cost will also integrate the social charges, the labor charges, and the depreciation rate of the equipment and productivity asset [15]. All these parameters were adjustable according to the economical standard of the area of the production. In order to study the virtual optimal mechanism, the mathematical model of the objective function relative to the various performance criteria is established [16]. Assuming that in the biomechanics of artificial limb, all the fingers contribute actively to accomplish if necessary each of the six grasping object modes retained by Pelletier and Vinet, Ruben, and Carrozza et al., taking into account the fact that the humanoid thumb mobility in particular among other fingers, the optimal design will be carried out on the base of minimization or maximization of single or a set of objectives function submitted to the various constraints [17–19]. Finally, the entire optimization process will be necessary to appreciate the influence of the said criteria on the prosthesis's human hand design. After the analysis of the mechanism consisting of the development of all the mathematical relations necessary to be summited to the optimization processes, for its synthesis, we will make the optimal synthesis of the said mechanism by reference to seven positions. Using the data relating to the thumb, the results obtained will be compared and discussed according to the state of art [20].

To mechanically simulate the different grasping mode of the object by an artificial hand, planar articulated mechanisms with one simple degree of freedom are generally recommended in hand prosthetic applications [21–25]. Based on this configuration, 1DOF four-crossed bar mechanism is considered in this study to design the thumb which is usually optimized by the means of transmission angle and energy consumed which have a significant effect on the mechanism design. To improve the use of these devices for the patients in need, new additional criteria will be modeled and integrated with the optimization process as objective functions. The first is the manufacturing cost, which would impact the affordability of the prosthesis by the amputees, and the second is the reliability of the setting mechanism and its effect on the prosthesis design. In the first approach, each criterion will be optimized individually and the three first criteria will be optimized simultaneously. Strength reliability and manufacturing cost will be considered individually, and finally, we will carry out the optimization of all the five criteria simultaneously [20].

## 2. Material and Methods

The thumb's mechanism description, its performance criteria, and its objective functions are presented in this section.

### 2.1. Thumb Finger Description

The thumb finger associated with the four-bar mechanism fit out with its driving system is depicted in Figure 1.

Figure 1 is made of a cable connected both to the driving link at the point *T*(*x*_*T*_, *y*_*T*_) and to the driving pulley at the point *C*(*x*_*C*_, *y*_*C*_) whose connection angle is *ρ*. The structure of thumb mechanism is added in the revised manuscript as Figure 2.

Table 1 defines the different parameters shown in Figure 1.

Freudenstein's relation [23–25, 28] between *θ*_1*i*_ and *θ*_2*i*_ at any mechanism position *i* is given by

(1) $$\begin{array}{c} k_{1}\cos\left(\theta_{1i}-\theta_{4}\right)+k_{2}\cos\left(\theta_{2i}-\theta_{4}\right)-k_{3}=\cos\left(\theta_{1i}-\theta_{2i}\right), \end{array}$$

where  *k*_1_ = *r*_4_/*r*_2_,  *k*_2_ = *r*_4_/*r*_1_, *k*_3_ = (*r*_1_^2^ + *r*_2_^2^ − *r*_3_^2^ + *r*_4_^2^)/(2*r*_1_*r*_2_), $r_{1}=\sqrt{P1^{2}+{\text{EXC}}^{2}}$, *θ*_1*i*_ = TP1_*i*_ − arctg(EXC/*P*1), *θ*_2*i*_ = *θ*_*A*_ + TP1_*i*_ + TP2_*i*_, $r_{1}=\sqrt{P1^{2}+{\text{EXC}}^{2}}.\sin\left(\text{THMP}-\text{arctg}\left(\text{EXC}/P1\right)\right)/\theta_{B}$, and $\theta_{B}=\text{arctg}\left(\sqrt{P1^{2}+{\text{EXC}}^{2}}.\sin\left(\text{THMP}-\text{arctg}\left(\text{EXC}/P1\right)\right)/\left(M1+\sqrt{P1^{2}+{\text{EXC}}^{2}}.\cos\left(\text{THMP}-\text{arctg}\left(\text{EXC}/P1\right)\right)\right)\right)$.

The values of some parameters in Equation (1) are similar to those used in [24] and are given in Table 2.

The design parameter value bounds of the thumb's mechanism are taken in [14] and are given in Table 3.

The vector *X* of the independent variables of the design is defined as

(2) $$\begin{array}{c} X={\left[x_{1},x_{2},x_{3},x_{4},x_{5},x_{6},x_{7},x_{8},x_{9}\right]}^{T}={\left[\theta_{A},r_{2},r_{3},r_{4},\theta_{4},t_{m},x_{T},y_{T},d\right]}^{T}, \end{array}$$

since the length of *r*_1_ is fixed and *θ*_*A*_ = *θ*_2*i*_ − (TP2_*i*_ + TP1_*i*_ + THMP).

In this study, the weight of the thumb mechanism was assumed to be negligible due to the dimensionless bars constituting the four-crossed bar mechanism used to model this artificial thumb [20].

### 2.2. Performance Criteria and Objective Functions of the Thumb Prosthesis Mechanism

The thumb prosthesis design is optimized by using the following five performance criteria:

- Least square structural error on the bending angle of the second phalanx should be minimized to ensure that the prosthetic finger should align at the prescribed positions
- Mechanical error on the bending angle of the second phalanx, due to dimensional tolerances and clearances on the articulations, should be minimized
- Maximum shaft driving torque should be minimized and able to counterbalance a grasping force applied at the end of the thumb finger
- Strength reliability of the mechanism should be maximized to ensure the mechanical strength during grasping, holding, or pinching operations
- Manufacturing cost of the mechanism should be minimized to evaluate its effect on the design variables

The objective function associated with the least square structural error on bending angle TP2 is defined as

(3) $$\begin{array}{c} f_{1}\left(x\right)=\frac{1}{6}\overset{7}{\underset{i=1}{\sum }}{\left(\theta_{2ic}-\theta_{2id}\right)}^{2}, \end{array}$$

where *θ*_2*id*_ = *x*_1_ + TP1_*i*_ + TP2_*i*_ is the desired angle and *θ*_2*ic*_ is the computed angle. It is also called mean square error, which describes the error, given in the form of least square function, describing the error observed between the computed value *θ*_2*ic*_ and the given value *θ*_2*id*_ of the bending angle between the palmer plan and the second phalanx TP2 of the thumb [14].

The objective function associated with the mechanical error on bending angle TP2 is defined as

(4) $$\begin{array}{c} f_{2}\left(x\right)=\frac{1}{6}\overset{7}{\underset{i=1}{\sum }}{\left(0.003\sqrt{2\left[{\left(\frac{\partial \theta_{2i}}{\partial r_{1}}r_{1}\right)}^{2}+\overset{9}{\underset{j=1}{\sum }}{\left(\frac{\partial \theta_{2i}}{\partial x_{j}}x_{j}\right)}^{2}\right]}\right)}^{2}. \end{array}$$

By assuming that the frictional forces at joints are negligible, the objective function associated with the maximum shaft driving torque is defined as

(5) $$\begin{array}{c} f_{3}\left(x\right)=\max\left(M_{P}\right)=\max\left(\frac{x_{9}M_{M}}{2\left(x_{7}\sin\beta +x_{8}\cos\beta \right)}\right), \end{array}$$

where  *β*  is the traction angle between the flexible cable on the driving system and the driving bar, *M*_*P*_ is the driving torque applied to the shaft, and *M*_*M*_ is torque reduced to point *M* of the driving bar. The objective function associated with the strength reliability of the mechanism is defined as

(6) $$\begin{array}{c} f_{4}\left(x\right)=R_{1}.R_{2}.R_{3}, \end{array}$$

where *R*_1_, *R*_2_, and *R*_3_ are the reliability of driven, junction, and driving bars, respectively [28, 29]. Since the prostheses are manufactured in very small sets, the manufacturing computer-aided design is appropriate for this purpose [30]. The manufacturing unitary cost of the *j*^th^ manufacturing operation on the *i*^th^ bar of the mechanism is

(7) $$\begin{array}{c} C_{u\left(ij\right)}=C_{p}+C_{Tm}-\frac{C_{S}}{N}+\pi L_{\left(ij\right)}D_{\left(ij\right)}\left[\left(\frac{C_{m}}{6\times 10^{4}\times V\times f}\right)+\left(\frac{C_{S}}{10^{3}\times f\times C^{-K}}V^{-K-1}\right)\right], \end{array}$$

where *C*_*p*_ = (*Ts*/*N*).(*Ap*/60), *C*_*T*_ = (*C*_*m*_/60).(*πL*_(*ij*)_.*D*_(*ij*)_/10^3^*V*.*f*), *C*_*Tm*_ = (*C*_*m*_/60)(∑_*j*=1_^3^*T*_*j*_ + *T*_*tm*_), and *C*_*o*_ = *C*_*S*_((*πL*_(*ij*)_.*D*_(*ij*)_/10^3^*f*.*C*^−*K*^)*V*^−*K*−1^ − (1/*N*))are the sum of the expenses related directly to the preparation, cutting duration, out of cutting time, and the cutting tool, respectively; *C*_*s*_ is the cost cutting tools; Ap is the global rate of exploitation of the preparation section, general expenses, and labor; *C*_*m*_ = *A* + *F* + *R* + *L* + *E* + *S* is hourly machine cost; *A*, *F*, *R*, *L*, *E*, and *S* are technical amortization, financial expenses, maintenance expenses and repair, expenses on local or on clutter, expenses on energy, and wage costs and social, respectively; *V*, *N*, *f*, and *k* are linear speed, mass production set, feed rate in turn/tooth, and Taylor constant function of material of the cutting tool, respectively; *D*_(*ij*)_ are the cutting tools used relatively at *i*^th^ bar and *j*^th^ manufacturing operation (milling cutter 2 cuttings ∅20, cutter 2 cuttings ∅6, drill ∅2, drill ∅4, piloting milling cutter to counter boring ∅2 × 6 and machining tapping *M*2); *L*_(*ij*)_ = *L*_*s*(*ij*)_ = *L*_*c*(*ij*)_ = *L*_*p*(*ij*)_ = *L*_*l*(*ij*)_ = *L*_*t*(*ij*)_ are the tool trajectories relative to the facing milling, lateral milling, drilling, counter boring, and tapping of the *i*^th^ bar of the mechanism and the *j*^th^ manufacturing operation, respectively; *T*_1_, *T*_2_, and *T*_3_ are the holes 1, 2, and 3, respectively, and  *Ts*  is execution duration allowed to the preparation of a set of workpiece. The manufacturing cost of the junction bar is

(8) $$\begin{array}{c} C_{3}=4C_{F}+\pi \left(L_{s\left(31\right)}D_{\left(31\right)}+L_{c\left(32\right)}D_{\left(32\right)}+L_{p\left(33\right)}D_{\left(33\right)}+L_{l\left(34\right)}D_{\left(34\right)}\right)\left[\left(\frac{C_{m}}{6\times 10^{4}V.f}\right)+\left(\frac{C_{S}}{10^{3}f.C^{-K}}V^{-K-1}\right)\right], \end{array}$$

where *L*_*s*(31)_ is the facing milling, *L*_*c*(32)_ is the lateral milling, *L*_*p*(33)_ is the drilling, and *L*_*l*(34)_ is the counterboring. The manufacturing cost of the driving bar is

(9) $$\begin{array}{c} C_{1}=4C_{F}+\pi \left(L_{s\left(11\right)}D_{\left(11\right)}+L_{c\left(12\right)}D_{\left(12\right)}+L_{p\left(13\right)}D_{\left(33\right)}+L_{l\left(14\right)}D_{\left(14\right)}\right)\left[\left(\frac{C_{m}}{6\times 10^{4}V.f}\right)+\left(\frac{C_{S}}{10^{3}f.C^{-K}}V^{-K-1}\right)\right], \end{array}$$

where *L*_*s*(11)_ is the facing milling, *L*_*c*(12)_ is the lateral milling, *L*_*p*(13)_ is the drilling, and *L*_*l*(14)_ is the counterboring. The manufacturing cost of the driven bar is

(10) $$\begin{array}{c} C_{2}=5C_{F}+\pi \left(L_{s\left(21\right)}D_{\left(21\right)}+L_{c\left(22\right)}D_{\left(22\right)}+L_{p\left(23\right)}D_{\left(33\right)}+L_{l\left(24\right)}D_{\left(24\right)}+L_{l\left(25\right)}D_{\left(25\right)}\right)\left[\left(\frac{C_{m}}{6\times 10^{4}V.f}\right)+\left(\frac{C_{S}}{10^{3}f.C^{-K}}V^{-K-1}\right)\right], \end{array}$$

where *L*_*s*(21)_ is the facing milling, *L*_*c*(22)_ is the lateral milling, *L*_*p*(23)_ is the drilling, *L*_*l*(24)_ is the counterboring, and *L*_*t*(25)_ is the tapping. The global manufacturing cost of the mechanism is

(11) $$\begin{array}{c} f_{5}\left(x\right)=C_{1}+C_{2}+C_{3}=13C_{F}+\pi M.LD, \end{array}$$

with

(12) $$\begin{array}{c} LD=\left(L_{s\left(11\right)}D_{\left(11\right)}+L_{c\left(12\right)}D_{\left(12\right)}+L_{p\left(13\right)}D_{\left(13\right)}+L_{l\left(14\right)}D_{\left(14\right)}+L_{s\left(21\right)}D_{\left(21\right)}+L_{c\left(22\right)}D_{\left(22\right)}+L_{p\left(23\right)}D_{\left(23\right)}+L_{l\left(24\right)}D_{\left(24\right)}+L_{l\left(25\right)}D_{\left(25\right)}+L_{s\left(31\right)}D_{\left(31\right)}+L_{c\left(32\right)}D_{\left(32\right)}+L_{p\left(33\right)}D_{\left(33\right)}+L_{l\left(34\right)}D_{\left(34\right)}\right), \end{array}$$

where *f*_5_(*x*) is in USD and the dimensions of all mechanism pieces are in millimeter [26]. The objective functions related to individual and multiobjective optimization are

(13a) $$\begin{array}{c} F_{1}=\left[f_{1}\left(x\right)\right], \end{array}$$

(13b) $$\begin{array}{c} F_{2}=\left[f_{2}\left(x\right)\right], \end{array}$$

(13c) $$\begin{array}{c} F_{3}=\left[f_{3}\left(x\right)\right], \end{array}$$

(13d) $$\begin{array}{c} F_{4}=\left[f_{4}\left(x\right)\right], \end{array}$$

(13e) $$\begin{array}{c} F_{5}=\left[f_{5}\left(x\right)\right], \end{array}$$

(13f) $$\begin{array}{c} f_{6}\left(x\right)=\left[f_{1}\left(x\right),f_{2}\left(x\right),f_{3}\left(x\right)\right], \end{array}$$

(13g) $$\begin{array}{c} f_{7}\left(x\right)=\left[f_{1}\left(x\right),f_{2}\left(x\right),f_{3}\left(x\right),f_{4}\left(x\right)\right], \end{array}$$

(13h) $$\begin{array}{c} f_{8}\left(x\right)=\left[f_{1}\left(x\right),f_{2}\left(x\right),f_{3}\left(x\right),f_{5}\left(x\right)\right], \end{array}$$

(13i) $$\begin{array}{c} f_{9}\left(x\right)=\left[f_{1}\left(x\right),f_{2}\left(x\right),f_{3}\left(x\right),f_{4}\left(x\right),f_{5}\left(x\right)\right]. \end{array}$$

Each of these multiobjective functions consists of a set of objective functions which are simultaneously optimized. The above functions expressed in terms of design variables are equality constraints *h*_*i*_(*x*) = 0 and inequality constraints *g*_*i*_(*x*) ≤ 0 according to the MATLAB optimization toolbox. The convergence criteria on the design variables *x*_*i*_, the objective functions *f*_*i*_(*x*), and the constraints *g*_*i*_(*x*) are, respectively, equal to 10^−7^, 10^−9^, and 10^−13^.

## 3. Results and Discussions

Three arbitrary points are chosen to conduct the optimization process to validate the results generated during the numerical simulations. Each objective function (known as least square structural error, mechanical error and strength reliability are dimensionless, maximum driving torque is expressed in N.mm, and manufacturing cost is expressed in USD) which is subjected to three equalities and eighteen inequality constraints is optimized by taking into consideration the design variable bounds in Table 3. Table 3 also gives the unit relative to each design variable. By using the optimum absolute value of every single function, the multiobjective optimizations *F*_6_(*x*), *F*_7_(*x*), *F*_8_(*x*), and *F*_9_(*x*) subjected to the same constraints are conducted. The optimization problem solved in this paper has a complex nature. We have five nonlinear objective functions subjected to all type of constraints and must be minimize simultaneously. There is no unique solution to the problem of multiobjective optimization of several objective functions expressed by mathematical expressions which are performance criteria. The selection of optimal solutions is based on Pareto-optimality conditions [31, 32]. A solution is called “pareto-optimal” if there is no other solution for which an improvement of an objective function does not lead to a degradation of at least one of the other functions. It is therefore important, for a problem of simultaneous minimization of several criteria, to generate the “pareto-optimal” solutions. It is what we achieve with “fgoalattain,” which solve multiobjective goal attainment problems. This method is implemented in “MATLAB” software using the “fgoalattain” minimization function. We have chosen the set of vector of the weighting coefficients *W* = absolute (goal) where absolute (goal) is the absolute value of the vector of the objectives set from individual optimization [33]. This condition guarantees the same percentage of achievement of the objectives set for all active objective functions [20]. The optimal design variables of the thumb mechanism are presented in Table 4.

Table 4 contains all the generated values of the design variables resulting from the optimization of each objective function and a set of coupled functions according to the optimization strategy adopted. The vectors of transversal, longitudinal, or angular dimensions of the virtual mechanisms are proposed at each optimum obtained. Individual optimization is represented by *F*1 to *F*5, and multiobjective optimization is represented by *F*6 to *F*9. The units of the various objective function are indicated in Table 5 as follows: *f*_1_(*x*) and *f*_2_(*x*) are in degree Celsius, *f*_4_(*x*) do not have unit, *f*_3_(*x*) is expressed in N.mm, and *f*_5_(*x*) is given in USD. The set of optimal design variable validated at each optimization problem corresponds to the situation where an objective function reaches a feasible solution on the computing solver, where all the constraints are satisfied with the lower and upper bounds. Figures 3–5 are plotted with the unit of *i* = 3, 4, and 5 in degree Celsius and with *i* = 1, 2, 6, 7, 8, and 9 in millimeters on *y*-axis. The optimal design variables versus individual and multiobjective optimization of thumb are presented in Figure 3.

Figure 3 helps to interpret the results relating to the optimal design variable, and it is associated with the optimization problem *Fi*. The *y*-axis shows the numerical values of the optimal design variable *xi*, and the abscissa axis is associated with the independent design variable. Table 5 presents the optimal values taken by the objective functions at the pareto-optimal solution for multiobjective optimization.

The other nonoptimal values calculated earlier when obtaining the optimal values of the functions to be optimized are removed from Table 5 for the reasons of clarity.  Figure 4 is plotted by using the partial data from Table 4 from the singular optimization.

Figure 4 facilitates the interpretation of the results relating to the optimal design variables relative to individual optimization. In essence, these variables are expressed as a function of the objective functions *f*_*i*_ relating to the various optimization problems *F*_*i*_ to be solved. Figures 3–5 are associated with a function *F*_*i*_, the *y*-axis shows the numerical values of the optimal design variable *x*_*i*_ with the unit of *i* = 3, 4, and 5 in degree Celsius and with *i* = 1, 2, 6, 7, 8, and 9 in millimeters as indicated in Table 3.  Figure 6 is associated with optimization problem Fi and the abscissa axis is associated with the functional transversal and longitudinal dimensions of the mechanism (xi). The units of the various objective functions are indicated in Table 5 as follows: *f*_1_(*x*) and *f*_2_(*x*) are in degree Celsius, and *f*_4_(*x*) do not have unit, while *f*_3_(*x*) is expressed in N.mm and *f*_5_(*x*) is given in USD. The optimal design variables versus multiobjective optimization of the thumb are presented in Figure 5.

Figure 5 is associated with the objective functions fi optimization problem Fi, the *y*-axis shows the numerical values of the optimal design variable xi, and the abscissa axis is associated with the variable design parameters.

Figure 5 is plotted based on the partial data from Table 4. The ordinate axis represents the optimal numerical values given by the design variables at the end of the process of simultaneous optimization of a set of coupled objective functions according to the strategy adopted. Moreover, Figure 3 helps to identify the behavior of individual design variables with respect to each simultaneous optimization problem.  Figure 4 which presents the behavior of each objective function versus the optimization problem is plotted by using Table 5.

Figure 6 demonstrates a proper understanding of the behavior of all the objective functions *f*_*i*_ relating to the optimization problems during the optimization process of each of the objective functions *F*_*i*_ relating to the different problems to be solved. The ordinate axis gives the values of the function *f*_*i*_ considered, and the abscissa axis shows all the functions *F*_*i*_ for all the resulting optimization strategies.  Figure 6 also gives a panoramic idea of the behavior of each objective function according to the optimization problem. The *y*-axis represents the optimal values taken by objective functions when an optimum is obtained at the end of the optimization process of the different optimization problems. Figures 4–6 show simultaneous optimization *F*_*i*_ of all the criteria confer on the thumb, with the same length of the fixed bar *r*_1_, the same thickness *x*_6_ = *t*_*m*_ of all the bars, and about the same diameter of the driving pulley. Two observations can be highlighted from the beginning of the manufacturing cost and reliability relating to the optimization process: the first is related to the reliability regarding all criteria being appreciably equal to the unit and the second observation is related to the minimum manufacturing cost, from which the largest design variable values are obtained. The manufacturing constraints such as geometrical and dimensional tolerances, accuracy (0.1 *μ*m), production set (*N*), cutting tool life span, and the shape of the workpiece guide the designer to choose the suitable manufacturing model cost parameters. The optimization process was conducted by varying three times the value of the stopping criteria as indicated at the end of the last paragraph of Section 2, to ensure the accuracy provided by the CNC machining process. The final results displayed at the end of optimization process are the optimal output, respecting all the constraints including manufacturing ones. The optimal objective function values from individual optimization were used as the weighting absolute goal to be achieved by the multiobjective “fgoalattain” solver. The steps where the system stop with the “nonfeasible” answer of the algorithm are cancelled and not validated for this study. The accuracy configures in the computing solver for design variable, objective function, and constraints are indicated in Section 2.2. From there, the precision observed on the results of Table 4 is justified and imposed to the manufacturer the used of computing-aided manufacturing to produce the part of this artificial mechanism.

The value of the optimal function obtained during the entire optimization process relative to the reliability of the whole mechanism is 0.9999, compared to 1 obtained by Ngale et al. [28], when only the driving bar was taken in consideration during the optimization processes. This difference of 0.1111 justifies the contribution of each bar in the reliability mathematical model. Furthermore, the multiobjective optimization showed that the mechanical reliability and the production cost included in any combination of the simultaneous optimization enabled the achievement of the same optimum variables design, though with some exceptions.

Earlier works from literature realized by Ngale et al. in 2003 and 2016, Lim et al. in 2018, and Tsamo et al. in 2020 on the prosthesis mechanism's optimization show that optimal design variables obtained from one single optimization to multiobjective optimization must be different to justify the contribution of the said performance criteria on the improvement of the design [24, 26, 27]. In this paper, the global manufacturing cost and the strength reliability of the whole mechanism are included in all combinations of the simultaneous optimization necessary to obtain the random optimum design variables. The optimal manufacturing cost generated from the numerical simulation is 501.0021 USD, for the thumb versus 961 USD for the thumb proposed by Ventimiglia [34] and 553 USD proposed by Choi et al., for one compliant finger, obtained by 3D printing [16]. The difference is 459.9979 USD with Ventimiglia price and 51.9979 USD with Choi et al. price. This difference is due to the inclusion of the power system, actuation, and miscellaneous component cost by Ventimiglia. The particularity of the cost generate on this study is that the design of the mechanism is based directly on the objective function modelled. The gap observed at the level of the price can be affected to numerous factors such as human factor error while evaluating empirical quantities, machine imprecision, labor charges, the depreciation rate of the equipment, and productivity assets which are included in the mathematical's manufacturing cost model of this study [35–37]. Otherwise, the simultaneous optimization *F*_*i*_ of all the criteria made it possible to reduce the standard deviation between all design variables. One notices that the virtual mechanisms of the fingers and the thumb are sensitive to each of the new performance criteria such as manufacturing cost and the strength reliability of the whole mechanism. The value of the optimal function obtained during the entire optimization process relative to the reliability  *F*_4_  is quite different with some exceptions of those obtained by Ngale and Vinet and Ngale who focused their study only on the reliability of the driving bar of the four-crossed bar mechanism [14, 20].

## 4. Conclusion

The paramount goal of this study was to optimize the thumb prosthesis's mechanism by taking into consideration the manufacturing cost model based on machining cost theory which took into detail the shape of the workpieces and the strength reliability of all the parts composing the entire mechanism. These criteria were added to those choosing from the state-of-the-art based on their popular contribution relative to the structure's design optimization. The virtual mechanisms of the thumb are sensitive to each of the new performance criteria employed. The value of the optimal function obtained during the entire optimization process relative to the reliability of the whole mechanism is 0.9999, compared to 1 obtained when only the driving bar was taken in consideration during the optimization processes. This difference of 0.1111 justifies the contribution of each bar in the reliability mathematical model. Furthermore, the multiobjective optimization showed that the mechanical reliability and the production cost included in any combination of the simultaneous optimization enabled the achievement of the same optimum variables design, though with some exceptions. It was found that the mechanical error has little influence on the design variables resulting from the simultaneous optimization. For the simultaneous optimization of all the criteria where it was integrated, its influence was reduced considerably because all the optimal values of the objective functions are lower than the value resulting from the individual optimization. The optimal manufacturing cost generated from the numerical simulation was 501.0021 USD, for the thumb versus 961 USD, and 553 USD for one compliant finger, obtained by 3D printing. The difference is 459.9979 USD and 51.9979 USD more than the price generated on this study. This difference is due to the inclusion of the power system, actuation, and miscellaneous component cost by Ventimiglia. The particularity of the cost generate on this study is that the design of the mechanism is based directly to the objective function modelled. The gap observed at the level of the price can be affected to numerous factors such as human factor error while evaluating empirical quantities, machine imprecision, labor charges, the depreciation rate of the equipment, and productivity assets which are included in the mathematical's manufacturing cost model of this study. Therefore, further studies in the biomechanics field could integrate the weight and the tribological phenomenon in the optimization processes of the mechanism to achieve the real design of these artificial devices.

## Figures and Tables

**Figure 1:** Schematic diagram of the thumb finger fit out with its driving system.

**Figure 2:** Structure of thumb finger mechanism without its driving system.

**Figure 3:** Optimal design variables versus individual and multiobjective optimization of thumb.

**Figure 4:** Optimal design variables versus individual optimization of thumb.

**Figure 5:** Optimal design variables versus multiobjective optimization of thumb.

**Figure 6:** Behavior of each objective function versus optimization problem.

**Table 1:** Designations of different parameters shown in Figures 1 and 2 [8, 20, 24–27].

Parameters	Designations
*P*	The applied force with an angle of *θ*_*P*_ to the axis of the corresponding phalanx
*F*_Tmax_	Maximum tension developed in the cable
*P*1, *P*2, *P*3	Lengths of proximal, middle, and distal phalanges (*P*3 = 0 for the thumb), respectively
*P*3′	Effective length of the distal phalanx, *P*3′ = 0 for the thumb
QM, AM, BA, and QB	Fixed, driving, junction, and input bar, respectively
TP1, *φ*, and *ψ*	Bending angles of phalanges with respect to the plane of the palm
TP2, TP3	Bending angles of *P*2 and *P*3 were measured from one phalange to another, respectively
*θ*_*P*_	Angle between force at the tip of the finger with the axis of the phalanx
*θ*_1_, *θ*_2_, *θ*_3_, and *θ*_4_	Angles of the phalanges of the mechanism with respect to a plane parallel to the plane of the palm
*Q*	Trapezometacarpal articulation
*M*1	Thumb metacarpal
*P*2′	Operative length of the second phalanx *P*2
TP1	Bending angle of *M*1 according to palmar plan
THMP	Bending angle of *P*1 according to *M*1 (fixed angle)
*θ*_*A*_	The angle between the second phalanx axis and the various links
*θ*_*B*_	The angle between *M*1 and the various links
*r*_1_	Length of the input bar, *r*_1_ = QB
*r*_2_	Length of junction bar, *r*_1_ = BA
*r*_3_	Length of driving bar, *r*_1_ = AM
*r*_4_	Length of the fixed bar, *r*_1_ = QM
DP1, DP2, and WR3	Diameters of phalanges *P*1 and *P*2 and width of links, respectively
EXC	Eccentricity
*d*	Pulley diameter
*t*_*m*_	Bar thickness

**Table 2:** Dimension values of thumb's mechanism [20, 24].

Parameters	Values
DP1	15 mm
DP2	13 mm
WR3	5 mm
*P*1	43.5 mm
*P*2	29 mm
*P*3′	0 mm
EXC	2 mm
*θ*_*P*_	90°
TP1_1_	18°
TP1_2_	29°
TP1_3_	40°
TP1_4_	51°
TP1_5_	61°
TP1_6_	73°
TP1_7_	84°
TP21	14.274°
TP12	18.027°
TP23	24.022°
TP24	32.142°
TP25	41.416°
TP26	55.649°
TP27	75.760°
TP3	30°
*P*	45 N
*F*_Tmax_	400 N

**Table 3:** Design parameter value bounds of thumb's mechanism [14].

Design variable's designation	*θ*_*A*_ (degree Celsius)	*r*_2_ (mm)	*r*_3_ (mm)	*r*_4_ (mm)	*θ*_4_ (degree Celsius)	*t*_*m*_ (mm)	*x*_*T*_ (mm)	*y*_*T*_ (mm)	*d* (mm)
Vector of design variable	*x*1	*x*2	*x*3	*x*4	*x*5	*x*6	*x*7	*x*8	*x*9
Min	87.115	5	72.550	5	360	0.794	10	-5	10
Max	82.063	15	74.994	7.5	380	1.588	20	5	17

**Table 4:** Thumb optimum design variables versus optimization problem.

	*F*_1_(ΔTP2) 10^−6^(°)	*F*_2_(ΔTP2)_Mech_ (°)	*F*_3_ *M*_MAX_ (N.mm)	*F*_4_ *M*_COST_ (US $)	*F*_5_	*F*6	*F*7	*F*8	*F*9
*x*_1_ (°)	65.0351	65.0354	56.9923	61.2194	87.3142	63.3855	82.1528	82.0630	78.1932
*x*_2_ (mm)	7.5493	7.5492	9.3495	7.2766	8.3944	5.9964	5.0942	5.0603	5.0603
*x*_3_ (mm)	73.5694	75.5937	77.6547	75.4232	7 1.6646	74.9943	36.9875	37.0354	37.0354
*x*_4_ (mm)	11.8156	11.8154	12.8802	11.2983	11.2842	9.5121	6.0577	6.0197	6.0197
*x*_5_ (°)	352.4660	354.6590	360.0000	35 1.668	346.5512	344.8354	375.7396	375.6806	375.6806
*x*_6_ (mm)	1 .0624	1.1157	1.2784	1.1414	1.0824	1.1362	0.8485	0.8517	0.8517
*x*_7_ (mm)	17.0718	17.0714	15.7538	15.0278	18.2923	15.0012	20.0003	20.0001	20.0001
*x*_8_ (mm)	5.0000	5.0000	-4.9873	5.0000	-0.2794	-4.9827	5.0002	5.0001	5.0001
*x*_9_ (mm)	15.0000	15.2874	17.0000	17.0000	14.5945	12.6336	10.0000	10.0000	10.0000

**Table 5:** Thumb optimization problem versus optimum objective function values.

F_i_(x)	f_1_(ΔTP2)10^−6^ (°)	f_2_(ΔTP2)10_Mech_ (°)	f_3_M_Max_ (N.mm)	F_4_	F_5_M_cost_ (USD)
*F*1	3133.4298	—	—	—	—
*F*2	—	347.5135	—	—	—
*F*3	—	—	1255.7342	—	
*F*4	—	—	—	0.9999	—
*F*5	—	—	—	—	499.1203
*F*6	3133.4125	21.6122	2172.2236	—	—
*F*7	3515.4463	16.2193	1821.1116	1.0000	—
*F*8	1656.9551	21.6162	2498.5664	—	494.8459
*F*9	3133.4018	12.4923	2943.7501	1.0000	495.2544

## Data Availability

The data used to support the findings of this study are included within the article.

## References

[1] Zollo L., Roccella S., Guglielmelli E., Carroza M., Dario P. (2007). Biomechatronic design and control of an anthropomorphic artificial hand for prosthetic and robotic applications. *IEEE/ASME Transactions on Mechatronics*.

[2] Gama E. N., Sánchez O. F. A. (2014). *Anthropomorphic robotic hands: a review, Ingeniería y Desarrollo*.

[3] Wang X. (2013). The optimization design of six-bar linkage mechanism. *Telkomnika*.

[4] Galal A. H., Mohammed A. A., Maha M. L. (2011). Optimal synthesis of a 4-bar simple toggle. *Journal of American Science*.

[5] Bullock I. M., Zheng J. Z., De La Rosa S., Guertler C., Dollar A. M. (2013). Grasp frequency and usage in daily household and machine shop tasks. *IEEE Transactions on Haptics*.

[6] Belter J. T., Segil J. L., Dollar A. M., Weir R. F. (2013). Mechanical design and performance specifications of anthropomorphic prosthetic hands: A review. *The Journal of Rehabilitation Research and Development*.

[7] Kawasaki H., Mouri T. (2019). Humanoid robot hand and its applied research. *Journal of Robotics and Mechatronics*.

[8] Vinet R., Lozac'h Y., Nicolas B., Drouin G. (1995). Design methodology for a multifunctional hand prosthesis. *Journal of Rehabilitation Research and Development*.

[9] Chang L. Y., Matsuoka Y. A Kinematic Thumb Model for the ACT Hand.

[10] Engdahl S. M., Breanne P. C., Brian K., Alicia D., Chestek C. A. (2015). Surveying the interest of individuals with upper limb loss in novel prosthetic control techniques. *Journal of Neuroengineering and Rehabilitation*.

[11] Tomoyuki K., Koji F., Akimoto N., Takashi M., Toru S., Atsushi O. (2018). A new method of measuring the thumb pronation and palmar abduction angles during opposition movement using a three-axis gyroscope. *Journal of Orthopaedic Surgery and Research*.

[12] Tang J., Zhang X., Zong-Ming L. (2008). Operational and maximal workspace of the thumb. *Ergonomics*.

[13] Akgun G. G., Kaplanoglu E., Cetin A. E., Ulkir O. (2018). Mechanical design of exoskeleton for hand therapeutic rehabilitation. *Journal of Research in Mechanical Engineering*.

[14] Haulin E. N., Vinet R. (2003). Multiobjective optimization of hand prosthesis mechanisms. *Mechanism and Machine Theory*.

[15] Dietrich R., Garsaud D., Gentillon S., Nicol M. (1986). *Précis méthode d’usinage*.

[16] Choi K. Y., Akhtar A., Bretl T. A compliant four-bar linkage mechanism that makes the fingers of a prosthetic hand more impact resistant.

[17] Pelletier M., Vinet R. (1985). *Les prothèses de la main. Recherche Bibliographiques, École Polytechnique de Montréal*.

[18] Ruben P. (2011). *The Effect of Joint Locks in under-Actuated Hand Prosthesis; Master Thesis*.

[19] Carrozza M. C., Dario P., Vecchi F., Roccella S., Zecca M., Sebastiani F. The CyberHand: on the design of a cybernetic prosthetic hand intended to be interfaced to the peripheral nervous system.

[20] Ngale E. H. (1999). *Critères de performance et optimisation des mécanismes d’une prothèse de la main, Thèse de Ph.D. en génie mécanique*.

[21] Guo G., Qian Q., Gruver W. A single-DOF multi-function prosthetic hand mechanism with an automatically variable speed transmission.

[22] Guo G., Zhang J., Gruver W. A. (1993). Optimal design of a six-bar linkage with one degree of freedom for an anthropomorphic three-jointed finger mechanism. *Proceedings of the Institution of Mechanical Engineers, Part H: Journal of Engineering in Medicine*.

[23] Ngale E. H., Lakis A. A., Vinet R. (2001). Optimal synthesis of a planar four-link mechanism used in a hand prosthesis. *Mechanism and Machine Theory*.

[24] Lim D., Georgiou T., Georgiou T., Bhardwaj A., O’Connell G. D., Agogino A. M. Customization of a 3d printed prosthetic finger using parametric modelling.

[25] Todorov T. S. (2015). Synthesis of Four bar Mechanisms as Function Generators by Freudenstein - Chebyshev. *Journal of Robotics and Mechanical Engineering Research*.

[26] Ngale E. H., Tsamo N. (2016). Manufacturing cost and strength reliability effects on the optimal design of hand prosthesis mechanisms. *International Journal of Engineering and Technical Research*.

[27] Tsamo N., Toko D. T., Talla P. K. (2020). Impact of mechanical reliability and production cost on the thumbs four crossed bar mechanisms. *International Journal of Engineering and Applied Sciences (IJEAS)*.

[28] Ngale E. H., Vinet R., Klim Z. (1998). Influence du matériau et de la fiabilité sur le design optimal des éléments de machines. *Proceedings CSME Forum*.

[29] Klim Z. (1995). *Fiabilité et maintenabilité des systèmes mécaniques*.

[30] Gonzalez P. (1993). Commande Numérique par calculateur. Tournage/Fraisage/Centresd’usinage. *Editions Casteilla*.

[31] Statnikov R., Matusov J., Statnikov A. (2012). Multicriteria engineering optimization problems: statement, solution and applications. *Journal of Optimization Theory and Applications*.

[32] Matusov L. B. (2020). On Reqularization and Vector Optimization of Machine Design Variables. *IOP Conference Series: Materials Science and Engineering*.

[33] Grace A. (2018). *Optimization Toolbox For Use with Matlab, User_s Guide*.

[34] Ventimiglia P. (2012). *Design of a Human Hand Prosthesis*.

[35] Camargo M., Rabenasolo B., Jolly-Desodt A.-M., Castelain J.-M. (2003). Application of the parametric cost estimation in the textile supply chain. *Journal of Textile and Apparel Technology and Management*.

[36] Wicek D., Dariusz W., Ivan K. (2019). Cost estimation methods of machine elements at the design stage in unit and small lot production conditions. *Management Systems in Production Engineering*.

[37] Ben-Arieh D. (2000). Cost estimation system for machined parts. *International Journal of Production Research*.

